# Screening and Analysis of Biomarkers in the miRNA-mRNA Regulatory Network of Osteosarcoma

**DOI:** 10.1155/2022/8055052

**Published:** 2022-03-15

**Authors:** Gang Han, Quanyi Guo, Nan Li, Wenzhi Bi, Meng Xu, Jinpeng Jia

**Affiliations:** Department of Orthopedics, The Fourth Medical Center of General Hospital of PLA, Beijing 100048, China

## Abstract

Osteosarcoma is a malignant disease, and few effective strategies can completely overcome the prognosis of these patients. This study attempted to reveal the key factors and related molecular mechanisms of osteosarcoma via excavating public microarray datasets. The data were obtained from the Gene Expression Omnibus (GEO) database; the differentially expressed miRNAs and differentially expressed genes were obtained in GSE69470 and GSE12685l, respectively; the target of miRNAs were predicted with the miRDIP database; the functions of the factors were analyzed and visualized by the David database and R language, respectively. Moreover, the protein-protein interaction network and miRNA-mRNA network were performed with the STRING database and Cytoscape software to identify the hub nodes in GSE69470 and GSE12685. The results showed that 834 DEGs were found in GSE12685 and 37 miRNAs were found in GSE69470. Moreover, the target of 37 miRNAs were enriched in PI3K/AKT, P53, Wnt/*β*-catenin, and TGF-*β* pathways and related with skeletal system development and cell growth. Besides, the miRNAs including miR-22-3p, miR-154-5p, miR-34a-5p, miR-485-3p, miR-93-5p, and miR-9-5p and the genes including LEF1, RUNX2, CSF1R, CDKN1A, and FBN1 were identified as the hub nodes via network analysis. In conclusion, this study suggested that the miRNAs including miR-22-3p, miR-154-5p, miR-34a-5p, miR-485-3p, miR-93-5p, and miR-9-5p and the genes including LEF1, RUNX2, CSF1R, CDKN1A, and FBN1 act as key factors in the progression of osteosarcoma.

## 1. Introduction

Osteosarcoma is a serious bone malignancy with a high tendency of aggressiveness and metastases, which has a high incidence in childhood [1, 2]. Statistically, more than 60% of patients with osteosarcoma are under 25 years old [3]. At present, surgery combined with neoadjuvant chemotherapy is the pillar for osteosarcoma treatment [4]. In recent ten years, the application of multiple radiotherapy and chemotherapy techniques and mature modern surgical skills have effectively changed the prognosis of patients [5]. With the current therapy strategies, a 5-year survival rate of patients has increased to 70% [6]. However, many patients still find it difficult to escape the bad outcomes in the long term. Although accumulating research has continually figured out the potential reasons of osteosarcoma development, the detailed mechanisms of osteosarcoma remain unclear, and deep research is urgently necessary.

MicroRNAs play important roles in the metabolic activities of cells via regulating the expression of proteins [7, 8]. Several reporters have indicated that the miRNA profile of osteosarcoma exhibits a high difference with the normal tissues, and some miRNAs have been identified as the hub nodes in regulating the malignant behavior of the tumor cells, such as rapid proliferation and high invasion [9]. For osteosarcoma, the miRNA profiles of patients also exhibit significant differences compared with normal people. Microarray analysis has been frequently used for revealing RNA profiles of diseases, which is useful for analyzing the related pathological mechanisms [10]. Some research has revealed the related molecular mechanism of some tumors via microarray analysis [11, 12].

This study aimed to analyze the miRNA profile and identify the key miRNAs of osteosarcoma via the GEO database, reveal the functions and potential regulation mechanisms of the miRNAs, and finally provide some novel references for osteosarcoma treatment.

## 2. Materials and Methods

### 2.1. Data Source

The microarray datasets of GSE12685 and GSE69470 were obtained from the GEO database (https://www.ncbi.nlm.nih.gov). The raw data of the datasets were downloaded with the packages of the R language including GEOquery, dplyr, and Limma.

### 2.2. Identification of Differentially Expressed Genes

All datasets were analyzed with the GEO2R tools of GEO, and the expressed matrix files of the datasets were obtained. For GSE12685, 11 clinical pathological samples of osteosarcoma tumor and 2 differential normal human osteoblasts were used to identify the DEGs. For GSE69470, the DEGs were analyzed in human osteosarcoma cell lines and four normal human cell lines including chondrocyte cells, mesenchymal stem cells, osteoblasts, and skeletal muscle cells. The genes with |logFC| > 2 and *P* < 0.05 were considered as the differentially expressed genes (DEGs).

### 2.3. Screening of Potential Targets of the miRNAs

The common genes in the differentially expressed miRNAs in the matrix files were selected and then used for the next analysis. For GSE69470, the common differentially expressed miRNAs in the matrix files are the osteosarcoma tumor cells and differentially normal human osteoblast cells, osteosarcoma tumor cells, and mesenchymal stem cells (MSCs). The potential targets of common miRNAs were predicted with the miRDIP database (https://ophid.utoronto.ca/mirDIP/). The genes with a high minimum score (top 5%) were selected for the targets of the common miRNAs. Moreover, the common genes of the matrices were screed and visualized with VENNY (https://bioinfogp.cnb.csic.es/tools/venny/index.html).

### 2.4. Kyoto Encyclopedia of Genes and Genomes (KEGG) Enrichment Analysis

A KEGG enrichment analysis was performed for investigating the related pathways of osteosarcoma. For GES12685, the DEGs were analyzed with KEGG enrichment. For GSE69470, the potential targets of differentially expressed miRNAs were used for KEGG enrichment analysis. The genes were annotated and analyzed by the David database (https://david.ncifcrf.gov/), and the related pathways in the results with a *P* value <0.05 were visualized with the R language.

### 2.5. Gene Ontology (GO) Enrichment Analysis

GO enrichment analysis was used to identify the molecular functions of genes. For GES12685, the DEGs were annotated by the David database, and then the related ENTREZID of genes were analyzed with the packages of the R language including clusterProfiler and org.Hs.eg.db. For the miRNAs, the targets of them were analyzed with GO enrichment. Finally, the related functions module with a *P* value <0.05 were visualized with the R language.

### 2.6. Network Analysis

The PPI network analysis was performed to identify the hub nodes of osteosarcoma. In brief, the common genes of the targets of the miRNAs in GSE69470 and the DEGs in GSE69470 were analyzed with the STRING database (https://cn.string-db.org/), and then visualized with Cytoscape software. For the miRNA-mRNA network, the connection of the differentially expressed miRNAs in GSE69470 and the DEGs in GES12685 were structured with Cytoscape. For the miRNA-mRNA network, the differentially expressed miRNAs in GSE69470 and their targets were visualized by Cytoscape software (3.4.0).

## 3. Results

### 3.1. Identification of miRNAs of the Datasets

The datasets were used to analyze the differentially expressed miRNAs. For GSE12685, 11 clinical pathological samples of osteosarcoma tumor and 2 healthy samples of normal human osteoblast were used to identify the DEGs, and 424 downregulated genes and 410 upregulated genes were found in osteosarcoma (Figures 1(c) and 2(c)). For GSE69470, the differentially expressed miRNAs were analyzed in human osteosarcoma cell lines and four normal human cell lines including chondrocyte cells, mesenchymal stem cells, osteoblasts, and skeletal muscle cells. Compared with the expression profiles of chondrocyte, osteoblasts, and skeletal muscle cells, 45 downregulated genes and 10 upregulated genes were found in human osteosarcoma cell line (Figure 1). Compared with the expression profile of human mesenchymal stem cells, 43 downregulated genes and 16 upregulated genes were found in human osteosarcoma cell lines (Figure 1). Moreover, 37 common miRNAs were found in the matrices of GSE69470.

### 3.2. Identification of the Targets of the Common miRNAs

To identify the key miRNAs in the development of osteosarcoma, the 37 common miRNAs including 30 downregulated miRNAs and 7 upregulated miRNAs were screened in the differentially expressed miRNAs of osteosarcoma cell lines compared with normal differential cells or mesenchymal stem cells (Figure 2(c)). 37 common miRNAs were screened in GSE69470, and 4037 potential targets were predicted by the miRDIP database. Moreover, 114 common genes were screened from the DEGs of GSE12685 and the targets of miRNAs in in GSE69470 (Figures 3(c) and 3(d)).

### 3.3. Functional Modules Analysis

To investigate the pathological mechanism of osteosarcoma, the targets of the screened miRNAs in GSE69470, the DEGs in GSE12685, and the common genes of them were analyzed with the KEGG enrichment. The DEGs in GSE12685 were associated with the extracellular matrix organization, regulation of vasculature development, skeletal system development, and so on (Figure 3(a)). For GSE69470, it was found that the targets of the screened miRNAs were involved in the skeletal system development, covalent chromatin modification, cell growth, and so on (Figure 3(b)). Moreover, it was found that the common genes were related with skeletal system development, regulation of cellular response to growth factor stimulus, regulation of cell growth, and so on (Figure 3(e)).

### 3.4. Pathways Analysis

To reveal the regulation mechanism of osteosarcoma, the related pathways of the factors in GSE12685 and GSE69470 were investigated with KEGG enrichment. The results showed that the DEGs in GSE12685 were related with the PI3K-AKT pathway, the Hippo pathway, the MAPK pathway, and microRNAs in cancer, P53 pathways, the Rap1 pathway, the TGF-*β* pathway, and so on (Figure 4(a)). The targets of the screened miRNAs in GSE69470 were connected with pathways in cancer, the PI3K-AKT pathway, the MAPK pathway, and microRNAs in cancer, the Rap1 pathway, the P53 pathways, the TGF-*β* pathway, and so on (Figure 4(b)). Moreover, it was also found that the common genes of the targets in GSE69470 and DEGs in GSE12685 were also involved in the PI3K/AKT pathway, the Hippo pathway, the MAPK pathway, and microRNAs in cancer, P53 pathways, the TGF-*β* pathway, and the Rap1 pathway (Figure 4(c)).

### 3.5. Network Analysis

To reveal the molecular mechanism of osteosarcoma, the targets of the differentially expressed miRNAs in GSE69470, the DEGs in GSE12685, and their common genes were analyzed with the STRING database, and then visualized by Cytoscape. The results showed that LEF1, RUNX2, CSF1R, PTPRD, VAV3, WIF1, BMP3, TFEC, FZD3, PTCH1, THBS1, CDKN1A, FBN1, TGFB1, and IGFBP3 had connections with miR-22-3p, miR-154-5p, miR-31-5p, miR-34a-5p, miR-485-3p, miR-93-5p, and miR-9-5p (Figure 5).

## 4. Discussion

Although considerable research has focused on finding effective therapeutic strategies for osteosarcoma treatment in recent years, the prognosis of patients has been significantly improved [13]. In this study, the differentially expressed miRNAs in GSE69470 and the DEGs in GSE12685 were analyzed to reveal the pathological mechanism of osteosarcoma. miRNAs dysfunction has been widely confirmed as the critical reason for cancer development. For osteosarcoma, several reporters have indicated that miRNA disorders promote the malignant behaviors of the tumor cells [13]. In this study, a significant difference in the miRNA profiles of normal cell lines and tumor cell lines was also found in the datasets. Moreover, 834 DEGs were identified in GSE12685. Considering the difference of BM-MSCs and differentiated bone cells in miRNA profiles, this study identified 37 common differentially expressed miRNAs in osteosarcoma cells.

miRNAs are characterized with targeting 3′-UTRs of mRNA to repress the translation process of the related proteins [14]. In this study, 43 downregulated DEGs and 91 upregulated DEGs in GSE12685 were related with 7 upregulated miRNAs and 24 downregulated miRNAs in GSE69470, respectively. The upregulated genes including LEF1, RUNX2, CSF1R, PTPRD, VAV3, WIF1, BMP3, TFEC, FZD3, and PTCH1 were found to be upregulated in osteosarcoma. Moreover, LEF1, RUNX2, CSF1R, VAV3, and FZD3 have been reported to take part in the development of cancer. Reduced LEF1 could enhance the sensitivity of breast cancer cells to resensitizing docetaxel, and LEF1 downregulation could also inhibit the growth of osteosarcoma cells [15]. RUNX2 has been identified as an oncogene, which could activate the PI3K/AKT pathways to promote the development of breast cancer, and RUNX2 has been identified as a biomarker for osteosarcoma development. Low-expressed CSF1R could impede the growth and metastasis of osteosarcoma cells though inactivating ERK signaling [16, 17]. Downregulated VAV3 could inhibit the angiogenesis of osteosarcoma, and inhibited FZD3 can also block the invasion and malignant growth of osteosarcoma cells [18, 19]. In this study, genes including THBS1, CDKN1A, FBN1, TGFB1, and IGFBP3 were found to be downregulated in tumor cell lines. However, only CDKN1A and FBN1 function as the inhibitors in caner progression. Decreased CDKN1A has been found in multiple tumor cells, and several studies have shown that IGFBP3 could effectively inhibit the malignant behaviors of cancer cells. For osteosarcoma, CDKN1A upregulation could inhibit the proliferation and cell cycle of the cells [20]. Reduced FBN1 is related with the high invasiveness and metastasis of osteosarcoma, and increased FBN1 could also inhibit the epithelial-mesenchymal transition of osteosarcoma cells [21]. Thus, this study suggests that the hub nodes LEF1, RUNX2, CSF1R, VAV3, FZD3, CDKN1A, and FBN1 are key factors in the progression of osteosarcoma.

This study confirmed that the targets of the differentially expressed miRNAs were related with PI3K/AKT, AMPK, Wnt/*β*-catenin, TGF-*β*, P53 pathways, and so on, and miR-22-3p, miR-154-5p, miR-31-5p, miR-34a-5p, miR-485-3p, miR-93-5p, and miR-9-5p were related with hub nodes. The study has indicated that miR-22-3p can inactivate the Wnt/*β*-catenin to inhibit the progression of via gastric cancer directly targeting BCL9 [22]. Increased miR-154-5p, miR-34a-5p, and miR-485-3p could also suppress the progression of osteosarcoma. [23]. The studies have indicated that both miR-34a-5p and LEF1 were related with the activity of Wnt/*β*-catenin pathways. Moreover, it has been verified that miR-34a-5p can directly target LEF1 to act as a cancer suppressor in esophageal squamous cells [24]. The miR-22-3p has been proved to suppress the activity of the PI3K/AKT pathways and thus inhibit the development of colorectal cancer [25]. CSF1R has also been found to boost the viability of T-cell lymphoma [26]. In this study, CSF1R was identified as a potential target of miR-22-3p, which suggests that the increased CSF1R induced by miR-22-3p downregulation is one of the reasons for osteosarcoma development. However, increased miR-31-5p has been found in osteosarcoma cells but has been proved to have inhibitor roles in osteosarcoma, which is inconsistent with the profile of GSE12685. Moreover, miR-93-5p may functions as an oncogene which takes part in the development of various tumors [27, 28]. The study showed that CDKN1A upregulation induced by miR-93-5p CDKN1A could block the TGF-*β* and thus increase the therapeutic effects of chemotherapy on small cell lung cancer cells [29]. miRNA-9-5p has been found to upregulate and activate PI3K/AKT pathways in osteosarcoma [30]. Besides, miR-485-3p has been also proved to be involved in the cancer development via regulating TGF-*β* pathways, and RUNX2 has been widely confirmed as the downstream factors of TGF-*β*. In this study, RUNX2 was identified as the potential target of miR-485-3p.

## 5. Conclusion

In summary, this study suggests the miRNAs including miR-22-3p, miR-154-5p, miR-34a-5p, miR-485-3p, miR-93-5p, and miR-9-5p and the genes including LEF1, RUNX2, CSF1R, CDKN1A, and FBN1 are the key factors in the progression of osteosarcoma.

## Figures and Tables

**Figure 1:** Volcano plots of differentially expressed factors in GSE69470 and GSE12685l. (a) The differentially expressed factors of human osteosarcoma cells and differentiated bone cells in GSE69470. (b) The differentially expressed factors of human osteosarcoma cells and mesenchymal stem cells in GSE69470. (c) The differentially expressed factor in GSE12685l.

**Figure 2:** Heat maps of differentially expressed factors in GSE69470 and GSE12685l. (a) The differentially expressed factors of human osteosarcoma cells and differentiated bone cells in GSE69470. (b) The differentially expressed factors of human osteosarcoma cells and mesenchymal stem cells in GSE69470. (c) The DEGs of GSE12685l. (d) The common differentially expressed miRNAs in the matrix files are the osteosarcoma tumor cells and differential normal human osteoblast cells and osteosarcoma tumor cells and mesenchymal stem cells (MSCs).

**Figure 3:** The modular functions of DEGs in the progression of osteosarcoma. (a) Module gene GO enrichment analysis of DEGs in GSE12685l. (b) Module gene GO enrichment analysis of the targets of the differentially expressed miRNAs in GSE69470. (c) The common genes of the downregulated DEGs in GSE12685l and the upregulated differentially expressed miRNAs in GSE69470. (d) The common genes of the upregulated DEGs in GSE12685l and the downregulated differentially expressed miRNAs in GSE69470. (e) Module gene GO enrichment analysis of the common genes.

**Figure 4:** The modular functions of DEGs in the progression of osteosarcoma. (a) KEGG enrichment analysis of DEGs in GSE12685l. (b) KEGG enrichment analysis of the targets of the differentially expressed miRNAs in GSE69470. (c) KEGG enrichment analysis of the common genes.

**Figure 5:** Network analysis of the differentially expressed factors in GSE69470 and GSE12685l. (a) The PPI network of DEGs in GSE12685l. (b) The PPI network of the targets of downregulated differentially expressed miRNAs in GSE69470. (c) The PPI network of the targets of upregulated differentially expressed miRNAs in GSE69470. (d) The miRNA-mRNA network of upregulated differentially expressed miRNAs and the related targets. (e) The miRNA-mRNA network of downregulated differentially expressed miRNAs and the related targets. (f) The miRNA-mRNA network of hub nodes (miRNA: yellow and target: green).

## Data Availability

The data to support the findings of this study are available on reasonable request from the corresponding author.
